# Comparison of High-Statin Therapy vs Moderate-Statin Therapy in Achieving Positive Low-Density Lipoprotein Change in Patients After Acute Coronary Syndrome: A Randomized-Control Trial

**DOI:** 10.7759/cureus.20710

**Published:** 2021-12-26

**Authors:** Chamithra D Rupasinghe, Theodosios Kantas, Rohail Sani, Natalia M Avendaño Capriles, Ramil dadabhoy, Afreenish Gul, Camilo Andrés Avendaño Capriles, Noman Khurshid Ahmed, Sohaib Tousif

**Affiliations:** 1 Internal Medicine, Manipal College of Medical Sciences, Pokhara, NPL; 2 Department of Surgery, General Athens Hospital, Athens, GRC; 3 Medicine, Shifa College of Medicine, Islamabad, PAK; 4 Medicine, Universidad del Norte, Barranquilla, COL; 5 Medical College, Ziauddin University, Karachi, PAK; 6 Internal Medicine, Ziauddin University, Karachi, PAK; 7 Foundations of Clinical Research (FCR) Program, Harvard Medical School, Boston, USA; 8 Internal Medicine, Aga Khan University Hospital, Karachi, PAK; 9 Medicine, Ziauddin University, Karachi, PAK

**Keywords:** moderate-statin therapy, high-statin therapy, cardiac, acute coronary syndrome, ldl

## Abstract

Introduction: Statin use in secondary prevention after acute coronary syndrome (ACS) can play an important role in enhancing clinical outcomes, this has been proven in several randomized trials. This study was conducted to compare the efficacy of moderate-intensity and high-intensity statins in controlling low-density lipoprotein (LDL) after ACS.

Methodology: A randomized control trial was conducted at the Cardiology Department of Liaquat National Hospital, Karachi, Pakistan, from July 2020 to September 2021. During admission, patients were either started on a high-intensity statin dose (rosuvastatin 20 mg) or moderate-intensity statin (rosuvastatin 10 mg) by a computer-generated allocation sequence. Patients were followed-up in the outpatient department (OPD) after 3 months, and a lipid profile at follow-up was obtained. The percentage of LDL change was determined on 3 months of follow-up.

Results: A total of 590 patients were enrolled in the study. Out of all participants enrolled, 334 (80.48%) completed the 3-month follow-up. The mean age of participants was 58.08 (+12.06) years. High-intensity statin therapy is positively associated with positive LDL change (adjusted odds ratio [AOR]=4.45, P-value=0.001).

Conclusion: Our data implies that high-intensity statin medication may be an initial therapeutic option to decrease LDL. However, future randomized clinical trials should corroborate these findings.

## Introduction

Statin use after acute coronary syndrome (ACS) can play an important role in enhancing clinical outcomes, and this has been proven in several randomized trials [1-2]. In patients with the established coronary arterial disease (CAD), current guidelines advise using statins, particularly high-intensity statin therapy, but this has not been implemented into clinical practice [3-4]. Studies have shown that the East Asian population has lower baseline low-density lipoprotein cholesterol (LDL-C), better statin responsiveness, and greater susceptibility to statin therapy side effects than the Western population [5]. Furthermore, a recent randomized trial in an East Asian population failed to demonstrate the incremental clinical effectiveness of high-intensity statin medication [6].

Because of genetic polymorphism, the levels of statin plasma and its metabolites are higher in Asians than Caucasians [7-8]. Many studies have reported no significant differences in outcome with high-intensity statins than with moderate-intensity statins in Asian patients, raising questions whether routine high-intensity statins are required [9-10]. However, one trial found that Asians who achieved a less modern LDL-C target of 70 mg/dl benefited from high-intensity statins [11].

In multiple randomized trials, high-intensity statins have consistently outperformed moderate-intensity statins for secondary prevention of adverse cardiovascular events [12]. As a result, the 2013 American College of Cardiology (ACA) or American Heart Association (AHA) guidelines on the treatment of blood cholesterol advises high-intensity statins for individuals with atherosclerotic cardiovascular disease, such as atorvastatin 40 or 80 mg and rosuvastatin 20 or 40 mg [13]. However, it is unclear whether the favorable effects of high-intensity statins are due to the statin intensity itself or the lower levels of LDL-C achieved by high-intensity statins compared to moderate-intensity statins. In Pakistan, no study compared the efficacy of moderate-intensity and high-intensity statin in controlling LDL. Thus, this study was conducted to compare the efficacy of moderate-intensity and high-intensity statins in controlling LDL after ACS.

## Materials and methods

Study design: A randomized control trial was conducted at the Cardiology Department of Liaquat National Hospital, Karachi, Pakistan, from July 2020 to September 2021.

Inclusion criteria: All patients aged 25 to 85 years admitted with acute ACS (either new onset or having another episode) were enrolled in the study and whose lipid profile samples were obtained within 24 hours of the onset of the ACS.

Exclusion criteria: Patients were excluded if they were contraindicated to rosuvastatin such as hypersensitivity reactions including rash, pruritus, urticaria, and angioedema or who developed serious adverse effects of rosuvastatin (rhabdomyolysis with and acute renal failure, myopathy, liver enzyme abnormalities) that was assessed using laboratory and clinical findings and previous history. Patients with acute liver disease were also excluded (assessed by persistent elevations of hepatic transaminase levels). Pregnant and lactating women and patients who were already on statin therapy were also excluded from the study.

Ethical approval for this study was obtained from the institutional review board of Liaquat University Hospital (IRB Number: LUH_2020_06_05).

Sample size and sampling technique

The sample size was calculated considering the proportion of patients achieving LDL-C level of ≤100 mg/dL, i.e., 71% [14], 95% CI, design precision of 5%, and lost to follow-up 20%. The total sample size calculated was 590: 295 in high-intensity statin and 295 in medium-intensity statin therapy. Participants were enrolled using a non-probability consecutive sampling technique.

Data collection

After enrollment, patients’ baseline data was collected through chart review in-hospital and patient interviews. We recorded age, gender, BMI, diagnosis, prior cardiovascular history, other comorbidities, smoking status, and diagnosis. According to the guidelines, there are no precise LDL-C cut-offs for commencing statin therapy in individuals aged greater and lesser than 75 years. A class-I recommendation is that all ACS patients begin statin medication, irrespective of their baseline LDL-C level [15]. The ultimate goal is to reduce LDL-C of greater than or equal to 50% from their untreated baseline [16]. We categorized the patients into two groups, including positive (if they achieved a reduction in LDL-C of greater than or equal to 50%) and negative (if they did not achieve a reduction in LDL-C of greater than or equal to 50%) [15].

During admission, patients were either started on a high-intensity statin dose (rosuvastatin 20 mg) or moderate-intensity statin (rosuvastatin 10 mg) by a computer-generated allocation sequence. During their stay in the hospital, patients were clinically monitored for the development of an allergic reaction upon initiation of rosuvastatin. Baseline liver function tests were also obtained during admission. For standardization, all patients had prescribed a single brand of rosuvastatin. On discharge from the hospital, patients and their attendants were educated about the medicine, dose, and side effects.

Compliance with medication was assessed by providing patients with a dose chart to fill in every day after taking medicines. Non-compliant patients are those who have not taken a statin for more than 7 days in a month (consecutively or sporadically). Patients with whom contact has not been established after 3 months were considered unfollowed. Patients who were lost to follow-up or did not adhere to medications were excluded from the final analysis. Patients were followed-up in the outpatient department (OPD) after 3 months, and a lipid profile at follow-up was obtained. The percentage of LDL change was determined on 3 months of follow-up.

Statistical analysis

We treated analysis as intent-to-treat: patients not adhering to treatment and permanently lost to follow-up were excluded. Baseline characteristics of patients were presented as percentages for categorical variables and mean for continuous variables. Two groups (medium-intensity and high-intensity statin) were compared using the chi-square test and t-test for categorical and continuous variables, respectively. To assess the impact of statin therapy on LDL change, multivariable logistic regression was used. P-value <0.05 was considered significant.

## Results

A total of 590 patients were enrolled in the study. Of all participants enrolled, 150 (25.42%) were unadhered to statin therapy, and 116 (19.66%) were lost to follow-up. The remaining 334 (80.48%) completed the 3-months follow-up, including 138 in the high-intensity statin group and 196 in the moderate-intensity statin group.

The mean age of participants was 58.08 (+12.06) years, the majority of participants were male (71.26%), 83.83% of participants had at least one comorbidity. Of all participants who completed a 3-month follow-up, 58.58% were adherent to statin therapy, as shown in Table 1. The most common morbidity found among participants included hypertension (72.86%), previous history of coronary artery disease (64.29%), and diabetes (56.43%), as shown in Table 2. Table 3 shows the characteristics of participants categorized based on study groups. No significant difference was found between the two groups in terms of baseline characteristics of participants (P-value>0.05).

**Table 1:** Baseline characteristics of participants *Mean (Standard deviation) BMI: body mass index; NSTEMI: non-ST-elevation myocardial infarction; STEMI: ST-elevation myocardial infarction

Variable	Categories	n(%)
Age*		58.08 (+12.06)
Gender	Male	238 (71.26)
	Female	96 (28.74)
Comorbidity	No	54 (16.17)
	Yes	280 (83.83)
BMI	Underweight	20 (5.99)
	Normal	110 (32.93)
	Overweight	133 (39.82)
	Obese	71 (21.26)
Group	Moderate-intensity statin	196 (58.68)
	High-intensity statin	138 (41.32)
Smoking status	Current smoker	44 (13.17)
	Ex-smoker	20 (5.99)
	Never smoker	270 (80.84)
Diagnosis	STEMI	214 (64.07)
	Non-stable angina	94 (28.14)
	NSTEMI	26 (7.78)

**Table 2:** List of comorbidities among study participants PCI: percutaneous coronary intervention; CLD: chronic liver disease; CKD: chronic kidney disease

Comorbidity	n (%)
Diabetes mellitus	158 (56.43)
Hypertension	204 (72.86)
Prior coronary artery disease	180 (64.29)
Prior PCI	84 (30.00)
Prior heart failure	74 (26.43)
Prior stroke	28 (10.00)
Hepatitis or CLD	8 (2.86)
CKD	50 (17.86)
Others	26 (7.78)

**Table 3:** Baseline characteristics categorized on the basis of study groups *Mean (Standard deviation) NSTEMI: Non-ST-elevation myocardial infarction; STEMI: ST-elevation myocardial infarction

Variable	Categories	Moderate-Intensity Statin n(%)	High-Intensity Statin n(%)	P-value
Age*		58.79 (11.45)	57.08 (12.84)	0.104
Gender	Male	136 (69.39)	102 (73.91)	0.368
	Female	60 (30.61)	36 (26.09)	
Comorbidity	No	26 (13.27)	28 (20.29)	0.086
	Yes	170 (86.73)	110 (79.71)	
BMI	Underweight	8 (4.08)	12 (8.70)	0.263
	Normal	64 (32.65)	46 (33.33)	
	Overweight	78 (39.80)	55 (39.86)	
	Obese	46 (23.47)	25 (18.12)	
Smoking Status	Current smoker	20 (10.20)	24 (17.39)	0.161
	Ex-smoker	12 (6.12)	8 (5.80)	
	Never smoker	164 (83.67)	106 (76.81)	
Diagnosis	STEMI	126 (64.29)	88 (63.77)	0.867
	Non-stable angina	56 (28.57)	38 (27.54)	
	NSTEMI	14 (7.14)	12 (8.70)	

Impact of statin therapy

First, a univariate analysis was done using the chi-square test of independence to assess the impact of high-intensity statin therapy on LDL change. Table 4 shows that the statin therapy is significantly associated with LDL change (P-value=0.001). Other variables significantly associated with positive LDL change included age of participant (P-value=0.001), comorbidity (P-value=0.002), smoking status (P-value=0.045), and diagnosis (P-value=0.004). Variables significantly associated with positive LDL change were included in the final model developed using multivariable logistic regression. The final model was composed of four independent variables and an outcome variable.

**Table 4:** Univariate analysis of factors associated with LDL change *Factors significant at P-value<0.25 ^Mean (Standard deviation) LDL: low-density lipoprotein; NSTEMI: non-ST-elevation myocardial infarction; STEMI: ST-elevation myocardial infarction

Variable	Categories	Negative LDL Change	Positive LDL Change	P-value
Age^		59.82 (11.97)	54.13 (11.35)	0.001*
Gender	Male	166 (71.55)	72 (70.59)	0.858
	Female	66 (28.45)	30 (29.41)	
Comorbidity	No	28 (12.07)	26 (25.49)	0.002*
	Yes	204 (87.93)	76 (74.51)	
BMI	Underweight	14 (6.03)	6 (5.88)	0.966
	Normal	76 (32.76)	34 (33.33)	
	Overweight	91 (39.22)	42 (41.18)	
	Obese	51 (21.98)	20 (19.61)	
Group	High-intensity statin	161 (69.40)	35 (34.31)	0.001*
	Low-intensity statin	71 (30.60)	67 (65.69)	
Smoking Status	Current smoker	26 (11.21)	18 (17.65)	0.045*
	Ex-smoker	18 (7.76)	2 (1.96)	
	Never smoker	188 (81.03)	82 (80.39)	
Diagnosis	STEMI	149 (64.22)	65 (63.73)	0.004*
	Non-stable angina	72 (31.03)	22 (21.57)	
	NSTEMI	11 (4.74)	15 (14.71)	

Table 5 shows the impact of high-intensity statin therapy on LDL change after adjusting with other independent variables. High-intensity statin therapy is positively associated with positive LDL change (adjusted odds ratio [AOR]=4.45, P-value=0.001). Increased age is negatively associated with positive LDL change (AOR=0.96, P-value=0.005). In addition, the odds of positive LDL change are 53% lower among patients with at least one comorbidity than patients without any comorbidity (AOR=0.47, P-value=0.031). Last, patients diagnosed with NSTEMI have higher odds of positive LDL change than patients diagnosed with STEMI (AOR=3.32, P-value=0.022).

**Table 5:** Impact of high-statin therapy on LDL change (multivariable logistic regression) LDL: low-density lipoprotein; AOR: adjusted odds ratio; CI: confidence interval; NSTEMI: non-ST-elevation myocardial infarction; STEMI: ST-elevation myocardial infarction

Variable	Categories	AOR	95% CI	P-value
Group	High-intensity statin	Reference		
	Moderate-intensity statin	4.45	2.63-7.55	0.001
Age		0.96	0.94-0.99	0.005
Comorbidity	No	Reference		
	Yes	0.47	0.24-0.93	0.031
Diagnosis	STEMI	Reference		
	Non-stable angina	1.48	0.78-2.49	0.225
	NSTEMI	3.32	1.18-9.29	0.022

## Discussion

In the current study on 334 patients with ACS, patients who received high-intensity statin had better LDL change than patients who received moderate-intensity statin. In previous studies, higher-intensity statin therapy showed better clinical outcomes than moderate-intensity statin therapy, but these studies particularly focused on the Western population [17-18]. As per the 2013 ACC or AHA guidelines, high-intensity statins need to be used for all patients with deemphasized targeting specific LDL-C levels and atherosclerotic cardiovascular disease (ASCVD) [16].

In previous randomized trials, statin medication with an absolute reduction in LDL-C showed consistent prognostic effects for primary and secondary prevention [2-3]. Additionally, the experimental and clinical data demonstrated the pleiotropic impacts of statins like antithrombotic activity, oxidative stress reduction, endothelial function enhancement, and anti-inflammatory activity [19].

After adjusting for potential confounding variables in the current study, high-intensity statin therapy provided incremental benefits over moderate-intensity statin therapy in patients with the ACS. In individuals with established CAD, a recently accepted guideline recommends using high-intensity statin treatment [16]. However, Asian patients have distinct clinical and genetic backgrounds than Westerners, so this advice may not be immediately applicable to them. A pharmacokinetic study also showed that statins have a more significant effect in East Asian patients than in Western patients, related to differences in statin pharmacokinetics [20]. The current study showed different findings than previous studies that did not find any significant differences between lower- and moderate-statin therapy related to clinical outcomes.

Stronger statins may be helpful in high-risk East Asian individuals, such as those with left main disease, multi-vessel disease, or diabetes [20]. According to current guidelines, stronger statins with target LDL cholesterol levels of 70 mg/dL or a 50% reduction if the baseline LDL cholesterol is between 70 and 135 mg/dL would be more appropriate in these patients [21]. Thus, even in Asian people, high-statin therapy could be useful in high-risk patients.

The benefits of high-intensity statin therapy are visible in the current study regarding reduction of LDL. Only after 8 to 12 months of treatment, the JAPAN-ACS research find that statin therapy significantly reduces coronary atherosclerosis [22]. According to a recent meta-analysis, high-intensity statin therapy does not result in plaque regression in ACS patients during the first 3 months; nevertheless, plaque regression occurs after 6-12 months and lasts for more than 12 months [23]. When comparing studies using high-intensity statin treatment to trials using moderate-statin treatment, subgroup analysis demonstrated more dramatic decreases in LDL-C and major adverse cardiovascular events (MACE) risk in the high-intensity statin group [24]. A personalized treatment strategy with high-dose statins has been proven to be more effective than LDL-C-based target approaches in preventing coronary heart disease events [25].

The current study has certain limitations. First, the study was conducted at only one center in Karachi; therefore, the findings of this study should be confirmed in other prospective clinical trials with long-term clinical follow-ups. Second, the current study included a population in Pakistan only; thus, it might not be possible to generalize our findings to other regions. Considering the current study results, it is important to carry out future studies in larger sample size and involve more study sites to assess whether high-statin therapy is effective enough to promote positive clinical outcomes.

## Conclusions

In the current study, the efficacy of high-intensity statin therapy was compared with moderate-intensity statin therapy among patients with ACS. LDL management is one of the important components of cardiac disease management and thus considering the benefits of high-intensity statin in reducing LDL levels among patients with ACS, high-intensity statin medication may be an initial therapeutic option to decrease LDL. However, future randomized clinical trials should corroborate these findings.
